The article "Evaluation and Correlation Analysis of Mental and Psychological Factors and Premature Ejaculation in Patients with Benign Prostatic Hyperplasia in Mobile Medical System" was retracted in 2023. Reasons: signs of a paper mill; suspected computer-generated content; unreliable results or conclusions; concerns about the data.

# Evaluation and Correlation Analysis of Mental and Psychological Factors and Premature Ejaculation in Patients with Benign Prostatic Hyperplasia in Mobile Medical System

**DOI:** 10.1155/2022/8260640

**Published:** 2022-04-23

**Authors:** Xiaohui Peng, Min Fu

**Affiliations:** Urology Surgery (Andrology), The First Hospital of Qinhuangdao, Qinhuangdao, 066000 Hebei, China

## Abstract

Chronic prostatitis is a very common and very difficult disease. Based on the mobile medical system, this paper carried out a correlation analysis on the psychological factors and the evaluation of premature ejaculation in patients with benign prostatic hyperplasia. The article first analyzes the application in the field of mobile medical and then introduces the prostate image segmentation method based on the geometric active contour model. The emergence of automatic organ tissue segmentation technology is timely; it can help clinicians save a lot of manual segmentation time and has better reversibility and objectivity, and the theory of curve evolution is analyzed. Finally, this paper introduces the experimental research object and purpose, makes a statistical analysis of the symptoms of benign prostatic hyperplasia, and compares the incidence of psychological symptoms in patients with prostatitis under different factors. The experimental results of this paper show that 90% of prostatitis patients have mild psychological problems, and 10% have moderate psychological problems. Among them, the main reason for the psychological disorder of patients is depression, for which we should strengthen the care for patients.

## 1. Introduction

Due to the development of the social economy and the improvement of people's living standards, substances ingested by humans such as ethanol in beverages lead in automobile combustion exhaust gas. And the living habits are formed due to the acceleration of modern rhythm and the intensification of social competition, such as using a scooter for a long time in a relatively stable life posture, such as using modern instruments or computers. All of them can lead to congestion and enlargement of the prostate, which in turn can lead to inflammation of the prostate. At the same time, poor living habits and dietary patterns may induce the occurrence of chronic prostatitis, such as prolonged sitting and heavy drinking, which can cause damage to the prostate. Therefore, people have carried out various scientific researches on the disease and deeply explored various factors that affect the disease, which has important practical significance for preventing prostate lesions and improving the quality of life of prostate patients.

Chronic prostatitis is a very common and very difficult condition. Prostatitis has completely different symptoms due to the differences in its causes and pathological changes, the physiological conditions of clinical patients, and the adaptability to bacterial infection. Many patients are not satisfied with the diagnosis, and even many physicians find it very difficult. After setbacks and disappointments, clinical patients often lack confidence in the disease, which ultimately leads to a failure to make a reasonable diagnosis. Based on the mobile medical system, this paper carried out a correlation analysis on the psychological factors and premature ejaculation assessment of patients with benign prostatic hyperplasia, in order to provide help for clinical treatment [1, 2].

The article "Evaluation and Correlation Analysis of Mental and Psychological Factors and Premature Ejaculation in Patients with Benign Prostatic Hyperplasia in Mobile Medical System" was retracted in 2023. Reasons: signs of a paper mill; suspected computer-generated content; unreliable results or conclusions; concerns about the data.

The innovation of this paper is reflected in, firstly, the application in the field of mobile medicine is analyzed, and then, the prostate image segmentation method based on the geometric active contour model is introduced. In this paper, the symptoms of benign prostatic hyperplasia and the incidence of psychological symptoms in patients with prostatitis under different factors were analyzed and compared.

## 2. Related Work

According to the research progress at home and abroad, different scholars also have a certain degree of cooperative research on mobile medicine and benign prostatic hyperplasia. Kim and Lee propose a personalized health document summarization system that provides reliable personal health-related summaries for general healthcare consumers via mobile devices. The system works by exploiting biomedical concepts, semantic types, and semantic relationships extracted from the Unified Medical Language System. It analyzes personal health records derived from mobile personal health record applications to generate personalized summaries from multiple online health documents [3]. Zhu et al. first summarized the development characteristics of mobile medical technology at home and abroad and then combined the field research data to study the application mode of mobile medical application in GDTS and analyzed its advantages and disadvantages. Finally, they proposed four measures to further develop GDTS mobile medical applications [4]. Xie et al. proposed an application architecture and framework for a new type of cooperative emergency medical service system. The system enables efficient communication of information between emergency command centers, ambulances, and hospital dispatch centers and enables doctors in ambulances to work collaboratively with specialists from the relevant departments of the hospital. Mobile applications based on the Android operating system are developed for convenience and flexibility. The system can help doctors shorten treatment time, improve service quality, and reduce harm to patients [5]. Singla et al. present the design and development of a fuzzy expert system (FES) to identify the current stage of chronic kidney disease. The proposed fuzzy rule-based expert system is developed with the help of clinical practice guidelines, databases, and knowledge of expert teams. It was observed that the system succeeded in 93.75% of the tests. The system supports physicians in evaluating patients for chronic kidney disease [6]. Khasunovich et al. assessed the decrease in bladder contractility in patients with benign prostatic hyperplasia (BPH). The experiment conducted a urodynamic investigation in 146 BPH patients, which included uroflowmetry and pressure flow studies. The results showed that 56.2% of BPH patients had decreased detrusor contractility [7]. Tuyet et al. proposed a new method for content-based medical image retrieval based on salient regions and deep learning. The proposed method consists of two stages: an offline task of extracting local object features and an online task of content-based image retrieval in a database. Their evaluation of the proposed method is based on precision and recall values. The dataset includes 5 sets of medical images with varying quality from low to high. By using the best medical image quality group, precision has an accuracy of 91.61%, and recall has an accuracy of 89.61% [8]. Sboev analyzes the stages of creation, testing and practical implementation of the modern organizational, and personnel structure of mobile medical teams and their function to meet the needs of the peaceful population of Moscow during the prehospital period in Moscow. Studies have shown that an organizational basis in the field of medical support for the population in emergencies can ensure the formation of mobile medical units with labor and material resources while maximizing the use of the internal reserves of regional healthcare [9]. However, these scholars did not analyze the correlation between the mental and psychological factors of patients with benign prostatic hyperplasia and the evaluation of premature ejaculation in the mobile medical system, but only discussed its significance unilaterally.

The article "Evaluation and Correlation Analysis of Mental and Psychological Factors and Premature Ejaculation in Patients with Benign Prostatic Hyperplasia in Mobile Medical System" was retracted in 2023. Reasons: signs of a paper mill; suspected computer-generated content; unreliable results or conclusions; concerns about the data.

## 3. Evaluation and Correlation Analysis Method of Mental and Psychological Factors and Premature Ejaculation in Patients with Benign Prostatic Hyperplasia in Mobile Medical System

### 3.1. Application in the Field of Mobile Medical

Mobile medical care is to provide medical services and information by using mobile communication technologies such as PDA, mobile phone, and satellite communication. Specifically in the field of mobile Internet, medical and health App applications based on mobile terminal systems such as Android and iOS are mainly used. At present, according to the difference of objects and purposes, there are six major application categories in the field of mobile medical care [10, 11]. They are health education, health hotline, diagnosis and treatment support, training and communication of medical workers, remote monitoring and remote data collection, disease spread tracking, etc., as shown in Figure 1. The social phenomenon of mobile medical care is embodied in. The advantages of “TD-LTE” high-definition, mobile, and wireless technology can help medical staff in ambulances to obtain clear and fast remote guidance through mobile high-definition video, so as not to miss the “golden half hour” of treatment. Community doctors bring mobile medical diagnostic equipment and can invite large hospitals and doctors for remote consultation at any time. Mobile healthcare has the following characteristics: making medical services “ready at hand”, “adding fuel” to the reform of public hospitals, and the next “gold mine” of the communication industry.

1. Health education and knowledge popularization: the application of education and health awareness in the field of mobile medical care is mainly to transmit massive health information from the source to the receiver through short messages [12–14]. In this type of application, text messages will be sent directly to the user's mobile phone, and the content will cover a variety of topics, including detection and treatment methods, medical services, and disease management. Moreover, short messages can penetrate into relatively remote areas, where the level of public health education is low, and medical resources such as medical clinics and medical staff are also relatively limited [15]
2. Health hotline: through a set of specific phone numbers, people can use their mobile phones to obtain more medical services, including telephone consultations, service complaints, medical facility information, medicines, medical equipment, and mobile medical clinics
3. Diagnosis and treatment support: the application of diagnosis and treatment support is mainly to provide suggestions on diagnosis and treatment of patients for medical workers in remote areas, such applications can provide mobile phone applications, such as medical decision tree systems, to help medical workers make diagnoses, and can also provide diagnoses directly to patients [16]. Such cases are often referred to as “telemedicine,” where a patient can send a photo of a wound or condition to a remote physician as a reference for diagnosis. Diagnosis and treatment support programs can greatly reduce the time cost for patients in remote areas to obtain timely treatment
4. Communication and training of medical workers: the application of communication and training of medical workers in the mobile medical project mainly refers to providing professional information and resources for medical workers through mobile devices, thereby improving their business level and improving their professional skills. It can effectively achieve the training goals of medical staff in remote areas [17, 18]. In addition, communication between different medical institutions can be strengthened through mobile devices, which can realize information sharing and improve resource utilization
5. Remote monitoring and remote data collection: remote monitoring through mobile devices can effectively track the health of patients and respond in a timely manner, which plays an obvious role in cases of acute exacerbation of chronic diseases. In the case of scarce medical resources, remote monitoring can provide an outpatient-like function for the treatment of patients, and medical staff can also track the health status of patients in time after they are discharged from the hospital. The application of remote data collection mainly takes advantage of the low cost of mobile medical care and the rapid information update. Policy makers and healthcare providers in a country, region, or even community need accurate data to evaluate the effectiveness of existing policies and programs and then to formulate new policy programs [19, 20]. Compared with traditional methods, the use of mobile devices for information collection and reporting can effectively reduce costs.  Figure 2 shows the mobile medical system
6. The spread and tracking of diseases and infectious diseases: if some infectious diseases are not detected in time, it is very likely that they will develop into large-scale infectious diseases, and the damage and loss will be immeasurable. Relying on the ability of mobile devices to quickly capture and transmit disease information, such large-scale disease outbreaks can be well avoided and effectively controlled [21, 22]

A notable contribution of mobile applications is reducing medical errors. In the process of patient care, there may be mistakes in the handover of nursing staff, as well as mistakes in the execution of drug distribution, drug validity management, and specimen collection. Mobile healthcare can help improve the problem of seeing a doctor. Since the start of the new medical reform, the demand and development potential of China's medical and health industry informatization is huge. Accelerating the promotion of medical and health informatization business and deepening the medical and health industry have become the focus of the industry. Mobile medical care is subject to certain limitations: the impact of Internet bandwidth limitations and the outdated equipment in primary hospitals are not suitable for us to carry out mobile medical care.

The article "Evaluation and Correlation Analysis of Mental and Psychological Factors and Premature Ejaculation in Patients with Benign Prostatic Hyperplasia in Mobile Medical System" was retracted in 2023. Reasons: signs of a paper mill; suspected computer-generated content; unreliable results or conclusions; concerns about the data.

### 3.2. Prostate Image Segmentation Based on Geometric Active Contour Model

As a science, medical imaging belongs to biological imaging and includes diagnostic imaging, radiology endoscopy, thermal imaging techniques for medical use, medical photography, and microscopy. In medical images, volume and contour inspection of organ tissue is a complex and time-consuming process. In radiation therapy planning, uncertainty and variability in organ margins may lead to suboptimal treatment of some patients. Therefore, the emergence of automatic organ tissue segmentation technology is timely; it can help clinicians save a lot of manual segmentation time and has better reversibility and objectivity [23, 24]. Although a large number of scholars have researched and summarized some suitable segmentation methods, the segmentation of medical images still brings challenges to us due to the problems of organ shape variability and low image contrast [25, 26].

Active contour models are an architecture for extracting object contour lines from 2D images that may contain noise. Active contour model is also known as snake model. A global division method uses the prior knowledge of the shape and size of objects mastered by people in real life practice and the division method of the entire graphic characteristics of objects. It is different from the traditional graph division method that utilizes the local characteristics of graphs and can more effectively reduce the erroneous segmentation caused by the separately used graph brightness, gradient, and texture information [27].

The basic principle of using active contour mode to achieve image separation is to set an initial contour curve near the edge of the target contour. Under the combined influence of internal energy (effectively controlling the elongation and distortion of the curve) and external force (image capability), the energy function of the curve is averaged, and the segmentation contour of the target figure is obtained at the same time. The mathematical definition of the active contour model is as follows. In the region of interest of image *H*(*a*, *b*), a continuous and closed parameterized curve *B*(*v*): *B*(*v*) = [*a*(*v*), *b*(*v*)], *v* ∈ [0, 1] is initially defined. Under the action of the image external force *D*_ext_(*B*(*v*)), the curve of *B*(*v*) continuously evolves along the normal direction until it reaches the high-frequency signal boundary of the object. The mathematical expression of the energy functional is:

(1) $$\begin{array}{c} \min D_{b}^{\left(B\left(v\right)\right)}=\tau \int_{0}^{1}{\left\|B^{`}\right\|}^{2}dv+\varphi \int_{0}^{1}{\left\|B^{``}\right\|}^{2}dv+\omega \int_{0}^{1}D_{\mathrm{ext}}\left(B\left(v\right)\right)dv. \end{array}$$

Among them, *τ*, *φ*, and *ω* are positive weighting factors, which are used to adjust the proportions of continuity energy, curvature energy, and image energy, respectively. To solve for the extremum of this energy functional, applying the Lagrangian Formula yields:

(2) $$\begin{array}{c} \tau B^{`}-\varphi B^{``}-\omega \nabla {\text{D}}_{\mathrm{ext}}=0. \end{array}$$

By introducing the time variable *s*, the evolution formula of the curve *B*(*v*, *s*) can be obtained:

(3) $$\begin{array}{c} \frac{\mu B\left(v,s\right)}{\mu s}=\rho B^{`}\left(v,s\right)-\varphi B^{``}\left(v,s\right)-\omega \nabla D_{\mathrm{ext}}. \end{array}$$

The first item is the bending force of the curve, which controls the bending degree of the curve *B*(*v*, *s*). The smaller the value, the easier it is to bend. The second term is the rigid force of the curve, which represents the weight of the points approaching each other, which controls the continuity of the curve *B*(*v*, *s*). The third term is the image force, which controls and promotes the contour curve to move closer to the object boundary [28]. Under the combined action of these three forces, how to choose the appropriate parameter size and how to define the external force of the image become the keys to the fast and accurate segmentation of the image by the active contour model. Compared with traditional image segmentation methods, the active contour model can be well coupled with prior shape knowledge and has good robustness for target contour extraction and tracking in specific regions. It can be widely used in medical image processing such as microscopic images, ultrasound images, CT, and MRI. Although the active contour model has a wide range of applications and strong processing capabilities, the segmentation work cannot be completed if the initial contour placement is unreasonable. At the same time, if the parameter settings of the internal and external force parameters of the parameter curve are uncomfortable, the curve evolution ability will also be weak, which is manifested as the curve concave and insufficient curve tension.

The article "Evaluation and Correlation Analysis of Mental and Psychological Factors and Premature Ejaculation in Patients with Benign Prostatic Hyperplasia in Mobile Medical System" was retracted in 2023. Reasons: signs of a paper mill; suspected computer-generated content; unreliable results or conclusions; concerns about the data.

Regarding the problem that the curve is prone to collapse when the image capability is not strong, the balloon force can be introduced from the traditional active contour simulation, and a distance correlation number is added to the original balance formula. The balance formula of the original balloon model is:

(4) $$\begin{array}{c} \frac{\mu B\left(v,s\right)}{\mu s}=\rho B^{`}\left(v,s\right)-\varphi B^{``}\left(v,s\right)+l_{1}m\left(v\right)-l\frac{\nabla D_{\mathrm{ext}}}{\left\|D_{\mathrm{ext}}\right\|}. \end{array}$$

Among them, *l*_1_ is the weighting factor of the balloon force, and *m*(*v*) is the unit normal vector of the curve *B*(*v*, *s*). The positive or negative value of *l*_1_ determines the properties of the balloon force. When *l*_1_ is positive, the balloon force drives the curve to expand outward; when *l*_1_ is negative, the balloon drives the curve to contract inward.

Based on the problem that the traditional active contour method has great requirements on the placement position of the initial curve contour and cannot converge on the concave edge of the object, a new concept of image force is given, and a gradient vector flow model is given [29]. This model solves the traditional image force with diffusion differential formula, and its dynamic evolution formula is:

(5) $$\begin{array}{c} \frac{\mu B\left(s\right)}{\mu s}=\rho B^{`}\left(s\right)-\varphi B^{``}\left(s\right)+P,\\ \min\left(ℵ\right)=\iint p\left(p_{a}^{2}+p_{b}^{2}+t_{a}^{2}+t_{b}^{2}\right)+{\left\|\nabla g\right\|}^{2}{\left\|P-\nabla g\right\|}^{2}dadb. \end{array}$$

Using the gradient descent method, the dynamic iterative formula of the diffusion formula can be obtained as follows:

(6) $$\begin{array}{c} p_{1}\left(a,b,s\right)=p\nabla^{2}p\left(a,b,s\right)-\left(p\left(a,b,s\right)-g_{a}\left(a,b\right)\left(g_{a}{\left(a,b\right)}^{2}+g_{b}{\left(a,b\right)}^{2}\right)\right),\\ t_{1}\left(a,b,s\right)=t\nabla^{2}t\left(a,b,s\right)-\left(t\left(a,b,s\right)-g_{a}\left(a,b\right)\left(g_{a}{\left(a,b\right)}^{2}+g_{b}{\left(a,b\right)}^{2}\right)\right). \end{array}$$

Among them, *p* is the regularization factor, *g* is the edge of the target image; usually, the gradient of the image is taken:

(7) $$\begin{array}{c} g={\left\|\nabla \left(J_{\theta }\left(a,b\right)*H\left(a,b\right)\right)\right\|}^{2}. \end{array}$$

*J*_*θ*_(*a*, *b*) is a Gaussian function with variance *θ*. The proposed gradient vector flow model solves the shortcomings of the traditional active contour model in the processing ability of the concave area of the object, but there are still problems such as slow boundary convergence and easy to fall into local minima.

### 3.3. Curve Evolution Theory

The curve evolution theory refers to the use of the two most important geometric basic parameters that characterize the properties of the curve—the curvature of the curve and the unit normal vector of the curve to explore the change of the properties of the curve with time. Curvature represents the bending ability of the curve. The unit normal vector represents the direction of the curve.

The article "Evaluation and Correlation Analysis of Mental and Psychological Factors and Premature Ejaculation in Patients with Benign Prostatic Hyperplasia in Mobile Medical System" was retracted in 2023. Reasons: signs of a paper mill; suspected computer-generated content; unreliable results or conclusions; concerns about the data.

Let the noncrossing closed curve be:

(8) $$\begin{array}{c} B\left(q\right)=\left(a\left(q\right),b\left(q\right)\right), \end{array}$$

where any value in *q* ∈ [0, 1], then the tangent vector of the curve is:

(9) $$\begin{array}{c} S\left(q\right)=\frac{B^{`}\left(q\right)}{{\left|B^{`}\left(q\right)\right|}^{2}}=\left(\frac{a^{`}\left(q\right)}{\sqrt{a`{\left(q\right)}^{2}+b`{\left(q\right)}^{2}}},\frac{b^{`}\left(q\right)}{\sqrt{a`{\left(q\right)}^{2}+b`{\left(q\right)}^{2}}}\right). \end{array}$$

The normal vector is:

(10) $$\begin{array}{c} M\left(q\right)=\left(\frac{-b^{`}\left(q\right)}{\sqrt{a`{\left(q\right)}^{2}+b`{\left(q\right)}^{2}}},\frac{a^{`}\left(q\right)}{\sqrt{a`{\left(q\right)}^{2}+b`{\left(q\right)}^{2}}}\right). \end{array}$$

Tangent vector is:

(11) $$\begin{array}{c} S\left(v\right)=\left(\frac{\left(da\left(v\right)/dq\right)}{\left(da/dq\right)},\frac{\left(db\left(v\right)/dq\right)}{\left(dv/dq\right)}\right)=\frac{B^{`}\left(q\right)}{{\left|B^{`}\left(q\right)\right|}^{2}}. \end{array}$$

Take the curve length *v* as the parameter.

The second derivative of the curve:

(12) $$\begin{array}{c} B^{``}\left(v\right)=S^{`}\left(v\right)=lM. \end{array}$$

Among them, *l* represents the curvature of the curve at this point, and the curvature at *B*(*q*) is defined as the rate of change of the horizontal angle *n* of the tangent at this point with the orientation length *v*. That is, NN is the derivative of the radius of the inscribed circle at that point [30].  Figure 3 is a schematic diagram of the tangent vector and the normal vector of the curve.

From the definition of curvature, we get:

(13) $$\begin{array}{c} l=\frac{b^{``}}{{\left(1+b{`}^{2}\right)}^{1.5}}=\frac{a^{`}\left(q\right)b^{``}\left(q\right)-b^{`}\left(q\right)a^{``}\left(q\right)}{{\left(a^{`}{\left(q\right)}^{2}+b^{`}{\left(q\right)}^{2}\right)}^{1.5}}. \end{array}$$

The derivation process is as follows:

(14) $$\begin{array}{c} dv=\sqrt{{\left(da\right)}^{2}+{\left(db\right)}^{2}}=da\sqrt{1+{\left(\frac{db}{da}\right)}^{2}}. \end{array}$$

The same can be obtained:

(15) $$\begin{array}{c} B^{``}\left(v\right)=l\left(\frac{-b^{`}}{\sqrt{1+b{`}^{2}}},\frac{1}{\sqrt{1+b{`}^{2}}}\right)=lM. \end{array}$$

Adding the time parameter *s* to the curve, the expression of the motion curve is:

(16) $$\begin{array}{c} B\left(q,s\right)=\left(a\left(q,s\right),b\left(q,s\right)\right). \end{array}$$

With the change of the time parameter *s*, the velocity formula of the curve motion is obtained:

(17) $$\begin{array}{c} \frac{\partial B\left(q,s\right)}{\partial s}=f\left(q,s\right). \end{array}$$

Among them, *f* is the moving speed of the curve, which is the vector sum of the speed of the curve in the normal direction and the tangent direction at the point.

The article "Evaluation and Correlation Analysis of Mental and Psychological Factors and Premature Ejaculation in Patients with Benign Prostatic Hyperplasia in Mobile Medical System" was retracted in 2023. Reasons: signs of a paper mill; suspected computer-generated content; unreliable results or conclusions; concerns about the data.

Therefore, the formula can be rewritten as:

(18) $$\begin{array}{c} \frac{\partial B\left(q,s\right)}{\partial s}=nS\left(q,s\right)+\varphi M\left(q,s\right). \end{array}$$

Since the velocity in the tangential direction of the curve does not change the geometric characteristics and shape of the curve, only the influence of the velocity in the normal direction can be considered, and the velocity formula of the curve motion can be simplified as:

(19) $$\begin{array}{c} \frac{\partial B\left(q,s\right)}{\partial s}=\varphi M\left(q,s\right). \end{array}$$

Among them, *A* is the velocity in the normal direction, and an appropriate function can be chosen to control the evolution of the contour boundary.  Figure 4 shows the medical image segmentation process.

Biomedical image segmentation is an important part of biomedical image processing, and the effectiveness of image segmentation directly affects the effectiveness of computer-aided diagnosis systems [31]. Although the latest biomedical image separation algorithms are mentioned, the generality of the algorithms is often affected due to the characteristics and complexity of biomedical image processing. The principles of medical image imaging are diverse, and the image quality and degradation models are also different, resulting in the diversity of medical image segmentation methods.

## 4. Evaluation of Mental and Psychological Factors and Premature Ejaculation in Patients with Benign Prostatic Hyperplasia in the Mobile Medical System and the Results of the Correlation Experiment

### 4.1. Object and Purpose of the Study

This research is now planned to explore the clinical manifestations of chronic prostatitis (NIH-CPSI) score and its symptom self-rating scale (SCL) and self-rating depression scale (SDS) score status, and compared with the general control group, the physical performance and psychological reaction characteristics of chronic prostatitis patients were further analyzed. After analyzing the relationship between psychotherapy and the severity, condition, number of treatments, and mental state of clinical symptoms, explain the relationship between them. After explaining the influence of psychological factors on the prognosis of chronic prostatitis, it is convenient to provide correct opinions on the prevention and treatment of chronic prostatitis. At the same time, after preliminary research on the relationship between psychology and the severity and prognosis of chronic prostatitis, it will finally provide help for clinical treatment.

The article "Evaluation and Correlation Analysis of Mental and Psychological Factors and Premature Ejaculation in Patients with Benign Prostatic Hyperplasia in Mobile Medical System" was retracted in 2023. Reasons: signs of a paper mill; suspected computer-generated content; unreliable results or conclusions; concerns about the data.

Thirty outpatients with chronic prostatitis in an andrology clinic were selected as the main research objects, and 30 healthy people with the same conditions who volunteered to study were randomly selected as the control group for comparative study.

### 4.2. Statistical Analysis of Symptoms of Benign Prostatic Hyperplasia

There are many studies on the pathogenesis of benign prostatic hyperplasia, but the etiology has not yet been elucidated. Probably due to a disturbed balance of epithelial and mesenchymal cell proliferation and apoptosis. Other related factors are androgens and their interactions with estrogens, interactions between prostate stroma and glandular epithelial cells, growth factors, inflammatory cells, neurotransmitters, and genetic factors. In the early stage of benign prostatic hyperplasia, due to compensation, the symptoms are not typical. With the aggravation of lower urinary tract obstruction, the symptoms gradually become obvious. Due to the slow progression of the disease, it is difficult to determine the time of onset. Patients with benign prostatic hyperplasia often have other chronic diseases because they are elderly patients. During the diagnosis, attention should be paid to the general condition of the patient, and detailed consultation, physical examination, and laboratory tests should be carried out, and attention should be paid to the functions of the heart, lung, liver, and kidney. The symptoms of dysuria combined with various examinations can confirm the diagnosis. The danger of benign prostatic hyperplasia lies in the pathophysiological changes caused by lower urinary tract obstruction. Its pathology varies greatly among individuals, and not all of them are progressive. Some lesions do not develop to a certain extent, so even if there are mild obstructive symptoms, surgery is not always required.

After the clinical treatment symptoms were analyzed by severity (NIH-CPSI), the two components of pain symptoms and voiding performance evaluations were added. The patients with prostatitis were divided into mild cases with 0~9 points, general degree with 10~18 points, and severe cases with 19~31 points. The results are shown in Table 1.

As can be seen from the above table, the number of patients with mild and severe chronic prostatitis was 12, accounting for 40% of all the tested persons; the number of patients with moderate severity was 14, accounting for 46.7% of all the tested persons; the number of severe cases was 4, accounting for 13.3% of all the subjects tested.

The article "Evaluation and Correlation Analysis of Mental and Psychological Factors and Premature Ejaculation in Patients with Benign Prostatic Hyperplasia in Mobile Medical System" was retracted in 2023. Reasons: signs of a paper mill; suspected computer-generated content; unreliable results or conclusions; concerns about the data.

Among the 30 chronic prostatitis patients surveyed in this survey, the average score of SCL indicates that from the overall level, the patient's self-feeling level is on a scale of 1 to 5. Each question of SCL is scored on a scale of 1 to 5, and it is estimated that the average range of each factor is about 1 to 5. The range is divided into three levels: level 1 indicates a relatively normal level of health; level 2 indicates mild to moderate problems; level 3 indicates moderate to severe psychological problems. Statistics are performed on the frequency distribution of the average factor scores within this grading region, as shown in Figure 5.

It can be concluded from the figure that from the overall level, the number of patients with SCL average score of 1-1.99 is the largest, 27 cases, accounting for about 90%; there were 3 cases with mild to moderate problems, accounting for about 10% of the total. Among the mild-to-moderate cases, the first factor was depression, with a total of 8 cases, accounting for 26.7% of all the tested persons; obsessive compulsion in 5 cases, accounting for 16.7%; somatization in 3 cases, accounting for 10%; anxiety in 2 cases, accounting for 6.7%; and diet and sleep in 4 cases, accounting for 13.3%. This also shows that most patients with chronic prostatitis have not reached the normal level of mental health, and only 10% of patients have mild to moderate problems. Most of the patients with mild to moderate symptoms showed depression, obsessive-compulsive disorder, somatization, anxiety disorders, and other disorders. Serious problems have not yet been detected, but may be due to the relatively small number of cases.

Among the 30 patients with chronic prostatitis in the research group, the number and percentage of SDS scores ≥ 50 and 20 single factor scores ≥ 3 are shown in Table 2 and Table 3.

It can be concluded from the table that the depression status of patients with chronic prostatitis ranks first in the morning and evening. 70% of the patients had symptoms of heaviness in the morning and lightness in the evening, followed by a decline in ability, and 43.3% of the patients had this feeling. Other factors with more scores include life emptiness, decision disorder, decreased libido, thinking disorder, decreased interest, hopelessness, feeling of uselessness, decreased appetite, sleep disorder, and easy tiredness; the average equivalent scores of these items are all ≥3 points.

Comparing the results of the SCL test between the chronic prostatitis patient group and the control group, the results showed that the positive items of the two groups of SCL were 35.23 and 25.91, respectively, and the difference was very obvious. However, most of the ten factors in the study group exceeded those in the control group, and the differences were more obvious, as shown in Figures 6 and 7.

The article "Evaluation and Correlation Analysis of Mental and Psychological Factors and Premature Ejaculation in Patients with Benign Prostatic Hyperplasia in Mobile Medical System" was retracted in 2023. Reasons: signs of a paper mill; suspected computer-generated content; unreliable results or conclusions; concerns about the data.

By *t* test, compared with the control group, the scores of paranoia factor and other factors were significantly different (*P* < 0.05); the scores of somatization, obsessive-compulsive disorder, depression, anxiety, hostility, mental illness, and other factors were also significantly different (*P* < 0.01).

According to the prostatitis symptom score, the patients were divided into three categories: mild, moderate, and severe. The SCL scores of the three types of patients are compared in Table 4.

Analysis of variance was performed on the table, and the following results were obtained: when the symptoms of chronic prostatitis were mild, moderate, and severe, there was a significant difference in the SCL positive items in mild patients and moderate and severe patients (*P* < 0.05).

### 4.3. Comparison of the Incidence of Psychological Symptoms in Patients with Prostatitis under Different Factors

The course of disease, symptoms, number of visits, and other factors were graded, and the SDS total score ≥ 50 was used as the defining standard. Comparison of the incidence of depressive symptoms (SDS) in patients with chronic prostatitis under different factors is shown in Figure 8.

As can be seen from the figure, according to the clinical symptom score of chronic prostatitis, it is divided into mild, moderate, and severe. The incidence of depressive symptoms was 46.2%, 47.1%, and 75% in patients with a disease course of 1 year, 1-2 years, and more than 2 years, respectively. There was a significant difference between the duration of the disease and the incidence of depressive symptoms (*P* < 0.01).

The course of disease, symptoms, number of visits, and other factors were graded, and the number of SCL positive items >42 items was used as the defining standard to compare the incidence of psychosomatic symptoms in patients with chronic prostatitis under different factors, as shown in Figure 9.

As can be seen from the figure, according to the clinical symptom score of chronic prostatitis, it is divided into mild, moderate, and severe, and the positive detection rate of SCL in patients is 53.8%, 60%, and 66.7%. The severity of clinical symptoms was comparable to that of normal SCL, and there was a significant difference (*P* < 0.05). For patients with a disease duration of 1 year, 1-2 years, and within 2 years, the positive detection rates of SCL were 38.5%, 70.6%, and 75%, respectively. The duration of the disease was comparable to the SCL score, and there was a very significant difference (*P* < 0.01).

The article "Evaluation and Correlation Analysis of Mental and Psychological Factors and Premature Ejaculation in Patients with Benign Prostatic Hyperplasia in Mobile Medical System" was retracted in 2023. Reasons: signs of a paper mill; suspected computer-generated content; unreliable results or conclusions; concerns about the data.

## 5. Discussion

Due to the vigorous development of mobile communication technology, mobile medicine has begun to become a hot spot in the academic and medical fields. Mobile medicine refers to the use of mobile communication technology and electronic equipment for medical business and information management. Its most important feature is that it realizes the most universal medical business services in a timely and anywhere manner. The mobile phone has laid an important cornerstone for the use of mobile information technology to support the development of medical services facing the public and has become an efficient business tool for real-time service, access, and storage of medical information. However, there are still certain challenges in the realization of medical services based on mobile devices, such as the limitations of the computing capabilities of mobile devices, data storage capabilities, and security and rights management issues. In addition, although current mobile medical applications and research tend to serve large clinics, medical institutions, etc., they seldom consider ordinary users and services such as a large number of specialized outpatient clinics, traditional Chinese medicine clinics, or pharmacies.

## 6. Conclusions

Among the large number of patients with chronic prostatitis encountered clinically, many patients are often accompanied by various mental illnesses. The main symptoms are dizziness, insomnia, dreaminess, forgetfulness, easy fatigue, decreased sexual function, premature ejaculation, depression, pessimism, panic, and so on. The possible reasons for its formation are mainly due to the lack of a good understanding of the disease of prostatitis, especially listening to the propaganda of some surrounding news media or exaggerating the complexity, which seriously disturbs or damages the physical and mental health of patients, causing patients to be uneasy, confused and disturbed panic psychology, or some patients also have the role of guilt psychology. If someone gets sick from unclean sexual behavior or temporary erectile dysfunction due to prostate cell disease, but when he is confused and disturbed at the same time, many unmarried people still masturbate before marriage. There are also common clinical manifestations of chronic prostatitis, and its treatment is complicated. Many patients have been treated for many times, have taken medicine many times, and have undergone physiotherapy and prostate treatment many times. However, the result is that the onset time is delayed and difficult to heal, and it has the characteristics of easy recurrence after monitoring. According to clinical statistics, slow nonbacterial prostatitis is eight times the bacterial disease prostatitis. Therefore, many patients are mentally anxious, have no confidence in the treatment of their own diseases and even become discouraged, and have many delusions and hallucinations and even suicide tendencies, resulting in various obstacles in the depths of the soul. However, this wrong psychological factor will also affect the recovery of chronic prostatitis and the improvement of the prognosis, aggravate the original disease, and even repeat the disease.

The article "Evaluation and Correlation Analysis of Mental and Psychological Factors and Premature Ejaculation in Patients with Benign Prostatic Hyperplasia in Mobile Medical System" was retracted in 2023. Reasons: signs of a paper mill; suspected computer-generated content; unreliable results or conclusions; concerns about the data.

## Figures and Tables

**Figure 1:** Main application categories of mobile medical.

**Figure 2:** Mobile healthcare

**Figure 3:** Schematic diagram of curve tangent vector and normal vector.

**Figure 4:** Medical image segmentation process.

**Figure 5:** Score frequency distribution of SCL total mean and each factor mean.

**Figure 6:** Comparison of SCL scores between patients with chronic prostatitis and healthy controls (1).

**Figure 7:** Comparison of the mean score of SCL between patients with chronic prostatitis and healthy controls (2).

**Figure 8:** Comparison of the incidence of depressive symptoms (SDS) in patients with chronic prostatitis under different factors.

**Figure 9:** Comparison of positive detection rates of SCL in patients with chronic prostatitis under different factors.

**Table 1:** Prostate inflammation score.

	Number	The proportion (%)
Mild	12	40
Moderate	14	46.7
Severe	4	13.3
Total	30	100

**Table 2:** Frequency and percentage of SDS total score and single factor score (1).

	Number of people	Percentage (%)		Number of people	Percentage (%)
Melancholy	4	13.3	Loss of libido	9	30
Morning heavy and evening light	21	70	Weight loss	2	6.7
Cry easily	1	3.3	Constipate	1	3.3
Sleep disorder	6	20	Palpitations	1	3.3
Loss of appetite	7	23.3	Tired easily	6	6.7

**Table 3:** Frequency and percentage of SDS total score and single factor score (2).

	Number of people	Percentage (%)		Number of people	Percentage (%)
Difficulty thinking	9	30	Difficulty deciding	11	36.7
Decreased ability	13	43.3	Sense of uselessness	9	30
Disturbed	3	10	Emptiness of life	11	36.7
Despair	9	30	Worthless	2	6.7
Irritable	2	6.7	Loss of interest	6	20

**Table 4:** Comparison of SCL positive items with different severity of clinical symptoms.

Degree of symptoms	Number of cases	Degree of symptoms	Mean difference	Standard deviation	*P*
Mild	12	Moderate	-0.7021	0.2601	<0.05
		Severe	-1.0198	0.3012	<0.01
Moderate	13	Mild	0.7021	0.2601	<0.05
		Severe	-0.3302	0.2801	>0.05
Severe	5	Mild	1.0198	0.3012	<0.01
		Moderate	0.3302	0.2801	>0.05

## Data Availability

The data that support the findings of this study are available from the corresponding author upon reasonable request.

The article "Evaluation and Correlation Analysis of Mental and Psychological Factors and Premature Ejaculation in Patients with Benign Prostatic Hyperplasia in Mobile Medical System" was retracted in 2023. Reasons: signs of a paper mill; suspected computer-generated content; unreliable results or conclusions; concerns about the data.

## References

[1] Elhoseny M., Ramírez-González G., Abu-Elnasr O. M., Shawkat S. A., Arunkumar N., Farouk A. (2018). Secure medical data transmission model for IoT-based healthcare systems. *Ieee Access*.

[2] Farouk A., Alahmadi A., Ghose S., Mashatan A. (2020). Blockchain platform for industrial healthcare: vision and future opportunities. *Computer Communications*.

[3] Kim G. W., Lee D. H. (2018). Personalised health document summarisation exploiting Unified Medical Language System and topic-based clustering for mobile healthcare. *Journal of Information Science*.

[4] Zhu W., Shen Y., Hui Z., Yang X., Hu K. (2018). Study of the application of mobile medical technology in construction of grading diagnosis and treatment system. *Zhongguo yi liao qi xie za zhi = Chinese journal of medical instrumentation*.

[5] Xie P., Tang Y., Xu L. (2017). Study on cooperative emergency medical service system and mobile app development. *International Journal of Internet Protocol Technology*.

[6] Singla J., Kaur B., Prashar D. (2020). A novel fuzzy logic-based medical expert system for diagnosis of chronic kidney disease. *Mobile Information Systems*.

[7] Khasunovich A., Amdiy R. E., Kuzmin I. V. (2011). Decrease of urinary bladder contractility in patients with benign prostate hyperplasia. *Urologicheskie Vedomosti*.

[8] Tuyet V., Binh N. T., Quoc N. K., Khare A. (2021). Content based medical image retrieval based on salient regions combined with deep learning. *Mobile Networks and Applications*.

[9] Sboev A. O. (2020). Mobile medical unit as a rational model of modern mobile medical formation operating in the metropolis in emergency situations. *Research and Practical Medicine Journal*.

[10] Xiao F., Ding W. (2019). Divergence measure of Pythagorean fuzzy sets and its application in medical diagnosis. *Applied Soft Computing*.

[11] Li X., Jianmin H., Hou B., Zhang P. (2018). Exploring the innovation modes and evolution of the cloud-based service using the activity theory on the basis of big data. *Cluster Computing*.

[12] Lo C. K., Chen H. C., Lee P. Y., Ku M. C., Ogiela L., Chuang C. H. (2019). Smart dynamic resource allocation model for patient-driven mobile medical information system using C4.5 algorithm - ScienceDirect. *Journal of electronic Science and Technology*.

[13] Zhang Y., Sun L., Song H., Cao X. (2014). Ubiquitous WSN for healthcare: recent advances and future prospects. *IEEE Internet of Things Journal*.

[14] Jiang Y., Song H., Wang R., Gu M., Sun J., Sha L. (2017). Data-centered runtime verification of wireless medical cyber-physical system. *IEEE Transactions on Industrial Informatics*.

[15] Bogdanov A. A., Chernykh A. V. (2020). Concept of the system of marine mobile medical complexes. *Marine Medicine*.

The article "Evaluation and Correlation Analysis of Mental and Psychological Factors and Premature Ejaculation in Patients with Benign Prostatic Hyperplasia in Mobile Medical System" was retracted in 2023. Reasons: signs of a paper mill; suspected computer-generated content; unreliable results or conclusions; concerns about the data.

[16] Kong H., Chen J. (2021). Medical monitoring and management system of mobile thyroid surgery based on internet of things and cloud computing. *Wireless Communications and Mobile Computing*.

[17] Taheri M., Pouresmaeili F., Omrani M. D. (2017). Association of ANRIL gene polymorphisms with prostate cancer and benign prostatic hyperplasia in an Iranian population. *Biomarkers in Medicine*.

[18] Lv Z., Qiao L. Analysis of healthcare big data.

[19] Meshram C., Ibrahim R. W., Obaidat M. S., Sadoun B., Meshram S. G., Tembhurne J. V. (2021). An effective mobile-healthcare emerging emergency medical system using conformable chaotic maps. *Soft Computing*.

[20] Metwaly A. F., Rashad M. Z., Omara F. A., Megahed A. A. (2014). Architecture of multicast centralized key management scheme using quantum key distribution and classical symmetric encryption. *The European Physical Journal Special Topics*.

[21] Raut S., Pardeshi K. (2017). Wireless medical surveillance system. *International Journal of Electronics Engineering Research*.

[22] Abulkasim H., Alsuqaih H. N., Hamdan W. F. (2019). Improved dynamic multi-party quantum private comparison for next-generation mobile network. *IEEE Access*.

[23] Lomotey R. K., Deters R. (2018). Middleware for mobile medical data management with minimal latency. *Information Systems Frontiers*.

[24] Hu M., Zhong Y., Xie S., Lv H., Lv Z. (2021). Fuzzy system based medical image processing for brain disease prediction. *Frontiers in Neuroscience*.

[25] Zhao Y., Li H., Wan S. (2019). Knowledge-aided convolutional neural network for small organ segmentation. *IEEE Journal of Biomedical and Health Informatics*.

[26] Yang Y., Lou G., Chen S., Guan S., Wang W., Yang B. (2017). Technical aspects of transurethral plasmakinetic enucleation and resection of the prostate for benign prostatic hyperplasia. *Minimally Invasive Therapy*.

[27] Prasetyo A. D. (2021). Ekspresi Hsa-miR-22-3p pada urin pasien benign prostate hyperplasia (BPH) sebagai biomarker non invasif. *BERITA BIOLOGI*.

[28] Molina N. M., Aristizábal A. F., Valencia J. G. (2020). Complication related factors in patients undergoing open simple prostatectomy due to benign prostate hyperplasia in a Colombian hospital. *Archivos Españoles de Urología*.

[29] Tian Y., Su Z. Y., Liu D. Y. (2020). Bladder outlet obstruction index alone is not reliable for the diagnosis of benign prostate hyperplasia. *National Journal of Andrology*.

[30] Krikovi Z., Simatovi M., Luki D., Stanojević A., Škrbić V., Janjić G. (2020). Frequency of common complications during treatment of patients with benign prostate hyperplasia. *Scripta Medica*.

The article "Evaluation and Correlation Analysis of Mental and Psychological Factors and Premature Ejaculation in Patients with Benign Prostatic Hyperplasia in Mobile Medical System" was retracted in 2023. Reasons: signs of a paper mill; suspected computer-generated content; unreliable results or conclusions; concerns about the data.

[31] Chakroun M., Zouari S., Saadi A. (2020). State of the art: open prostatectomy for benign prostate hyperplasia: should we avoid it in all cases?. *La Tunisie Médicale*.

